The article "Sialyl Lewis X as a predictor of skip N2 metastasis in clinical stage IA non-small cell lung cancer" was published in 2013. Journal: World J Surg Oncol.

# Sialyl Lewis X as a predictor of skip N2 metastasis in clinical stage IA non-small cell lung cancer

**DOI:** 10.1186/1477-7819-11-309

**Published:** 2013-12-06

**Authors:** Hiroaki Komatsu, Shinjiro Mizuguchi, Nobuhiro Izumi, Kyukwang Chung, Shoji Hanada, Hidetoshi Inoue, Shigefumi Suehiro, Noritoshi Nishiyama

**Affiliations:** 1 Department of Cardiovascular Surgery, Osaka City University Graduate School of Medicine, 1-4-3 Asahi-machi, Abeno-ku, Osaka 545-8585, Japan

**Keywords:** Non-small cell lung cancer, Sialyl Lewis X, Skip N2, Surgery, Prognosis

## Abstract

**Background:**

Radical segmentectomy has been performed for small-sized non-small cell lung cancer (NSCLC). However, underestimation of mediastinal lymph node metastasis in the absence of hilar or interlobar metastasis (skip N2) affects surgical strategy. Our aim was to investigate preoperative and intraoperative predictors of skip N2 in clinical stage (c-stage) IA NSCLC.

**Methods:**

From 1998 to 2011, 279 patients (155 men and 124 women) with c-stage IA NSCLC (230 pN0, 17 pN1, 12 skip N2, 20 non-skip N2) underwent systematic lobectomy (R0 resection) at our institute. We compared preoperative serum concentrations of carcinoembryonic antigen, cytokeratin 19 fragment, sialyl Lewis X (SLX), and pre- and intraoperative clinicopathological features of pN0 and skip N2 patients. Receiver operator characteristic (ROC) curve analysis was performed to distinguish between the two patient groups.

**Results:**

The 5-year survival rate of skip N2 patients was 78.6%, higher than that of non-skip N2 patients (44.9%), and not significantly different than that of pN0 (86.7%) or pN1 patients (82.4%). The mean serum SLX concentration in skip N2 patients (28.0 U/ml) was elevated compared to that in pN0 patients (22.9 U/ml). In ROC analysis of SLX, the area under the curve was 0.710, and the optimal cut-off value was 21.4 U/ml (sensitivity, 91.7%; specificity, 51.7%). In multivariate analysis, SLX was an independent predictor of skip N2 in patients with c-stage IA NSCLC (odds ratio, 9.43; *p* = 0.006).

**Conclusions:**

Skip N2 metastasis is common in patients with c-stage IA NSCLC with high serum SLX, and lobectomy with complete dissection of hilar and mediastinal lymph nodes should remain the standard surgical procedure for these cases.

## Background

Lung cancer is the leading cause of cancer-related deaths worldwide [1]. The treatment of non-small cell lung cancer (NSCLC) depends on the stage of the disease [2]. Lobectomy with radical lymph node dissection remains the standard initial therapy for patients with stage I, II, and IIIA NSCLC [3,4], but limited resection has also been performed for early stage NSCLC. The Lung Cancer Study Group performed a pivotal study comparing limited resection (segment or wedge) with lobectomy for clinical stage (c-stage) IA NSCLC and found inferior overall survival and three times the local recurrence rate in the limited resection group [5]. Radical segmentectomy has been performed for small-sized (tumor diameter ≤3 cm) c-stage IA NSCLC [6-8]. In reported studies there was no significant difference in overall 5-year survival rates between patients undergoing segmentectomy compared to lobectomy (75.0 to 89.8% and 81.0 to 84.0%, respectively) [6-9]. In a separate study, Whitson *et al*. reported that lobectomy conferred superior unadjusted overall and cancer-specific 5-year survival compared with segmentectomy [10]. Thus, the issue of surgical strategy remains controversial. A phase III study is underway in Japan to evaluate overall survival of patients with small-sized (tumor diameter ≤2 cm) peripheral NSCLC treated with segmentectomy versus lobectomy (JCOG0802/WJOG4607L) [11].

The surgical indication for radical segmentectomy must include negative hilar and mediastinal lymph node metastases. If any diseased lymph node is found, segmentectomy should be converted to standard lobectomy. In some reports, segmentectomy was performed in patients with NSCLC (tumor diameter ≤2 cm) negative for lymph node metastasis, as confirmed by frozen-section intraoperative examination [12,13]. However, N2 lymph node metastasis without N1 hilar or interlobar lymph node involvement (skip N2 metastasis) might be overlooked if segmentectomy is performed with frozen-section examination of hilar and interlobar lymph nodes only. It has been reported that among 275 patients with c-stage IA NSCLC who were scheduled to undergo radical segmentectomy, 15 patients (6%) had pathologically confirmed N1 or N2 disease, and 4 of these (27%) had skip N2 metastasis [14]. Recently, intraoperative sentinel-node biopsy has been performed using new methods, such as isotope [14,15] or indocyanine green fluorescence [16] to avoid overlooking skip N2 metastasis. Patients with skip N2 have a better prognosis than non-skip N2 patients (overall 5-year survival rate, 34.4 to 41.0% and 14.0 to 24.0%, respectively) when treated with lobectomy and hilar and mediastinal lymph node dissection [17-22]. Therefore, accurate preoperative prediction of lymph node involvement is very important in planning adequate surgical resection. Our aim was to investigate the preoperative and intraoperative predictors of skip N2 and to recommend appropriate surgical resection in small-sized (tumor diameter ≤ 3 cm) c-stage IA NSCLC.

## Methods

Two hundred seventy-nine patients (155 men and 124 women, mean age 66.2 years) with c-stage IA (tumor diameter ≤3 cm) NSCLC underwent pulmonary resection (R0) at Osaka City University Hospital from January 1998 to December 2011. The surgical procedure performed was potentially curative complete resection by systematic lobectomy in combination with hilar and mediastinal lymph node dissection (over ND2a-1). When lymph node metastases in lymph nodes number 10, 11, and 12 were suspected intraoperatively, these lymph nodes were examined by frozen section. Patients with preoperative chemotherapy or radiation therapy were excluded from the study. Pathological diagnoses were performed by at least two pathologists in our hospital according to the criteria of the World Health Organization [23], and stages were classified according to the tumor, metastasis, node (TMN) classification of the International Union Against Cancer [24]. Chest and abdominal computed tomography (CT), magnetic resonance imaging (MRI) of the brain, bone scintigraphy, and positron-emission tomography (PET) were performed to examine the distant metastasis. If CT revealed a mediastinal lymph node with a short axis-length over 10 mm, mediastinal staging was performed using video-assisted thoracotomy, fine-needle aspiration with bronchoscopy, or PET. The sites of the N1 and N2 lymph nodes were determined based on primary tumor location according to the International Association for the Study of Lung Cancer using the new lymph node map for NSCLC [25]. Skip N2 metastases were defined as N2 lymph node metastases without N1 node involvement. Histopathologic evaluations were done by microscopic examinations of hematoxylin and eosin staining. Proportion of ground-glass opacity (GGO) area was calculated as follows:

$$\begin{array}{l} \left(\left(\mathrm{Area}\;\mathrm{on}\;\mathrm{lung}\;\mathrm{window}\;‒\;\mathrm{Area}\;\mathrm{on}\;\mathrm{solid}\;\mathrm{window}\right)\right)\\ \;\left(/\mathrm{Area}\;\mathrm{on}\;\mathrm{lung}\;\mathrm{window}\right)\times 100. \end{array}$$

Preoperative serum concentrations of carcinoembryonic antigen (CEA), cytokeratin 19 fragment (CYFRA21-1), and sialyl-Lewis X (SLX) were measured in each patient.

### Institutional review board approval and informed consent

This study was approved by the ethics committee at Osaka City University Graduate School of Medicine. Written informed consent was received from all patients.

### Statistical analysis

All statistical analyses were performed using GraphPad Prism, version 5 (GraphPad Software, San Diego, CA, USA) and JMP, version 9 (SAS Institute, Cary, NC, USA). Differences in serum levels of CEA, CYFRA21-1, and SLX were analyzed for statistical significance using a nonparametric test (Mann–Whitney *U*-test). Receiver operating characteristic (ROC) curve analysis was used to determine the optimal cutoff point and the sensitivity and specificity of each tumor marker to distinguish skip N2 patients from patients without pathological lymph node metastasis (pN0). The area under the ROC curve (AUC) was calculated. Statistical significance of the associations between skip N2 and various clinicopathological variables was evaluated using univariate analysis and multivariate logistic regression analysis. Survival curves were calculated from the day of surgery to death or to final follow up using the Kaplan-Meier method, and differences in survival curves were assessed with the log-rank test. *P*-values <0.05 were considered statistically significant.

## Results

### Postoperative survival of patients with different pathological N factors

The 279 patients with NSCLC included 230 patients without pathological lymph node metastasis (pN0), 17 patients with hilar or interlobar lymph node metastasis (pN1), 12 patients with skip N2 metastasis, and 20 patients with non-skip N2 metastasis. Table 1 shows pathological stages of patients based on each pathological N factor. The median postoperative observation time was 47 months (range 2 to 148 months). The overall 5-year survival rates for patients with pN0, pN1, skip N2, and non-skip N2 were 86.7%, 82.4%, 78.6%, and 44.9%, respectively (Figure 1). The prognosis of skip N2 patients was significantly better than that of non-skip N2 patients (*P* = 0.018). There were no significant differences between the prognoses of skip N2 and pN0 or pN1 patients (*P* = 0.336, *P* = 0.700, respectively).

**Table 1:** Pathological stages of patients based on each pathological N factor

	**Number of patients**			
	**Pathological N0**	**Pathological N1**	**Skip N2**	**Non-skip N2**
Pathological stage				
IA/IB	189/31	0/0	0/0	0/0
IIA/IIB	0/4	17/0	0/0	0/0
IIIA	6	0	12	20

**Figure 1:** **Kaplan-Meier curves for postoperative overall survival of 230 pathologic (p)N0 patients, 17 pN1 patients, 12 skip N2 patients, and 20 non-skip N2 patients.** The prognosis of skip N2 patients was significantly better than that of non-skip N2 patients (*P* = 0.008). There was no significant difference between the prognosis of skip N2 and pN0 or pN1 patients (*P* = 0.801, *P* = 0.985, respectively). pN0: pathological N0; pN1: pathological N1.

### Distributions of serum CEA, CYFRA21-1, and SLX in pN0 and skip N2 patients

To avoid underestimating skip N2 metastasis with frozen-section examination of only hilar and interlobar lymph nodes, clinical and surgical features of pN0 and skip N2 patients were compared. Table 2 shows the mean serum concentration of CEA, CYFRA21-1, and SLX in pN0 and skip N2 patients. Serum concentrations of CEA and CYFRA21-1 were not significantly different between the two groups (*P* = 0.196, *P* = 0.936, respectively). As shown in Figure 2, serum concentration of SLX rose with increasing pathological N factor. The serum SLX levels in skip N2 patients (mean 28.0 U/mL) and non-skip N2 patients (mean, 33.6 U/mL) were significantly higher than in pN0 patients (mean, 22.9 U/mL; *P* = 0.015, *P* = 0.001, respectively). There was no significant difference between the serum SLX levels of pN1 (mean 25.1 U/mL) and pN0 patients (*P* = 0.226). The ROC curve of SLX concentration to distinguish skip N2 patients from pN0 patients is shown in Figure 3. The AUC was 0.710. The calculated optimal cutoff point for serum SLX level was 21.4 U/mL (Youden index = 0.433). The sensitivity of this cutoff was 91.7% (11 of 12 skip N2 patients), and the specificity was 51.7% (109 of 211 pN0 patients). ROC curve analysis of CEA levels was also performed. The AUC was 0.611, the optimal cutoff point was 2.8 ng/mL, and the sensitivity and specificity were 91.7% and 37.3%, respectively. There was no significant difference between the AUC of SLX and CEA (*P* = 0.227).

**Table 2:** Serum concentrations of CEA, CYFRA21-1, and SLX in pN0 and skip N2 patients

	**Number of patients**		**Mean serum level (95% CI)**		***P*-value**
	**Pathological N0**	**Skip N2**	**Pathological N0**	**Skip N2**	
CEA (ng/mL)	230	12	5.3 (4.5, 6.0)	5.4 (3.5, 7.4)	0.196
CYFRA21-1 (ng/mL)	219	12	1.4 (1.3, 1.6)	1.8 (0.6, 2.9)	0.936
SLX (U/mL)	211	12	22.9 (21.7, 24.1)	28.0 (23.5, 32.6)	0.015
CEA: carcinoembryonic antigen; CYFRA: cytokeratin 19 fragment; SLX: sialyl Lewis X					Mann-Whitney *U*-test

**Figure 2:** **Percentile distribution of serum sialyl Lewis X (SLX) concentrations in pathological (p)N0, pN1, skip N2, and non-skip N2 patients with clinical stage IA non-small cell lung cancer (NSCLC).** Each box contains the variable distribution between the 25th and 75th percentiles, with median value indicated with a line in the box. The bars extending above and below the box indicate the 90th and 10th percentiles, respectively. The mean SLX concentration was significantly higher in the skip N2 patients compared to that in the pN0 patients (*P* = 0.015).

**Figure 3:** **Receiver operating characteristic curve for serum sialyl Lewis X (SLX) in pathological (p)N0 and skip N2 patients.** The area under the curve (AUC**)** = 0.710. The calculated optimal cutoff point for serum SLX concentration was 21.4 U/mL (Youden index = 0.433), and the sensitivity was 91.7% (11 of 12 skip N2 patients), whereas the specificity was 51.7% (109 of 211 pN0 patients).

### Clinicopathological features of 12 skip N2 patients

Table 3 shows clinicopathological features of 12 skip N2 patients according to age, sex, tumor side, tumor location, histology, tumor size, proportion of GGO, distance from tumor to pleura on CT, serum concentration of SLX, lymph vessel invasion (ly) factor, venous invasion (v) factor, pathological pleural invasion (pPL) factor, and site of skip N2 metastasis. Of 12 patients with skip N2, 10 (83.3%) were positive for ly factor, and 5 (41.7%) were positive for v factor, whereas among pN0 patients, only 20.2% were positive for ly factor and 3.8% for v factor (*P* <0.001). On preoperative CT, eight of twelve skip N2 patients had peripheral lung cancers located close to the pleura (distance ≤5 mm). Six patients (50%) had lung cancer in the lower lobes; of these, three had skip metastasis to subcarinal lymph nodes and three had skip metastasis to upper mediastinal lymph nodes. By contrast, all six patients with lung cancer in the upper lobes had skip metastasis to upper mediastinal lymph nodes. In relation to the site of skip N2 metastasis, nine patients (75%) had single-station disease, and three patients (25%) had multi-station disease.

**Table 3:** Clinicopathological features of 12 skip N2 patients

**Pt. no.**	**Age/sex**	**Side**	**Location (lobe)**	**Histology**	**Tumor size (mm)**	**Proportion of GGO (%)**	**Distance to pleura (mm)**	**SLX (U/mL)**	**ly**	**v**	**pPL**	**Site of skip N2**
1	73/M	Rt	Upper	Sq	15	19	4	36.2	+	-	0	No. 2R, 4R LN
2	34/F	Rt	Upper	Ad	16	68	13	27.4	+	-	0	No.4R LN
3	70/F	Rt	Upper	Ad	21	47	30	21.4	+	+	0	No.2R, 4R LN
4	62/F	Rt	Upper	Ad	14	24	28	13.1	+	-	0	No. 4R LN
5	71/M	Rt	Lower	Ad	30	9	0	40.2	-	-	0	No. 7 LN
6	61/F	Rt	Lower	Ad	24	27	0	32.8	+	+	1	No. 7 LN
7	60 M	Rt	Lower	Ad	24	23	0	29.0	+	+	0	No.2R, 4R LN
8	62/F	Lt	Upper	Ad	20	72	5	23.6	+	+	1	No. 5 LN
9	81/M	Lt	Upper	Sq	27	13	0	24.5	+	-	2	No. 5 LN
10	63/M	Lt	Lower	Ad	15	38	0	28.0	+	-	0	No. 5 LN
11	60/M	Lt	Lower	Ad	23	7	14	27.0	-	+	0	No. 7 LN
12	57/F	Lt	Lower	Ad	20	3	0	33.0	+	-	0	No. 5 LN

Pt. no., patient number; M,male; F, female; Rt, right; Lt, left; Ad, adenocarcinoma; Sq, squamous cell carcinoma; GGO, ground-glass opacity; distance to pleura, measured on computed-tomography; SLX, sialyl Lewis X; ly, lymph vessel invasion factor; v, venous invasion factor; pPL, pathological pleural invasion factor; No. 2R, upper paratracheal lymph node; No. 4R LN, lower paratracheal lymph node; No. 5 LN, subaortic lymph node; No. 7 LN, subcarinal lymph node.

### Clinical and surgical features of pN0 and skip N2 patients

To reveal preoperative and intraoperative predictive factors for skip N2, we compared pN0 and skip N2 patients, looking for underestimation of nodal factors based on intraoperative hilar or interlobar lymph node examination. Table 4 lists the clinical and surgical features of 230 pN0 patients and 12 skip N2 patients according to age, sex, tumor side, tumor location, histology, tumor differentiation, tumor diameter, sPL factor, serum SLX concentration, and serum CEA concentration. Univariate analysis revealed that skip N2 was significantly associated with elevated serum SLX concentrations (odds ratio = 9.91; *P* = 0.007). There were no significant differences between the two groups in other clinical or surgical features. Results of multivariate analysis show that SLX was the only independent predictor of skip N2 metastasis in patients with c-stage IA NSCLC (odds ratio = 9.43; *P* = 0.006).

**Table 4:** Clinical and surgical features of 230 pathological (p)N0 patients and 12 skip N2 patients

	**Number of patients**		**Univariate**	**Multivariate**		
	**pN0**	**Skip N2**	***P*-value**	***P*-value**	**Odds ratio**	**95% CI**
Age						
Mean ± SD	66.5 ± 10.2	62.8 ± 11.4	0.268^a^			
Sex						
Male	121	6	1.000	NA	NA	NA
Female	109	6				
Side						
Right	131	7	1.000	NA	NA	NA
Left	99	5				
Location						
Upper/Middle lobe	151	6	0.353	NA	NA	NA
Lower lobe	79	6				
Histology						
Ad	192	10	1.000	NA	NA	NA
Sq/AdSq	38	2				
Tumor differentiation						
Well/moderate	181	7	0.146	0.361	1.80	0.49, 6.13
Poor	49	5				
Tumor diameter (cm)						
≤2	113	6	1.000	NA	NA	NA
>2	117	6				
sPL factor						
sPL0	141	6	0.547	NA	NA	NA
sPL1-3	89	6				
SLX (U/mL)						
≥21.4	121	11	0.007	0.006	9.43	1.75, 175
<21.4	109	1				
CEA (ng/mL)						
≥2.8	143	11	0.060	0.077	4.78	0.87, 89.2
<2.8	87	1				
Ad: adenocarcinoma			Fisher’s exact test	Multivariate logistic regression analysis		
Sq: squamous cell carcinoma			^a^Mann-Whitney *U*-test			
AdSq: adenosquamous carcinoma						
sPL factor: surgical pleural invasion factor						
CI: confidence interval						

## Discussion

Radical segmentectomy with systematic lymph node dissection has been performed for small-sized NSCLC [7,8,14,15]. When intraoperative frozen-section examination of hilar or interlobar lymph node reveals metastasis, we believe segmentectomy should be converted to standard lobectomy. The question of whether radical segmentectomy allows adequate lymph node dissection remains controversial, because the mean number of dissected lymph nodes with segmentectomy is significantly lower than with lobectomy [7]. Intraoperative frozen-section examination of hilar or interlobar lymph can detect pN1 or non-skip N2 disease, which leads to appropriate surgical resection. However, underestimation of skip N2 due to the difficulty of examining all mediastinal lymph nodes intraoperatively leads to challenges in choosing the appropriate surgical procedure. In a study on intraoperative sentinel lymph node identification, Kim *et al*. reported that five of forty c-stage I NSCLC patients (12.5%) had mediastinal sentinel lymph nodes without hilar lymph node involvement [26]. One mechanism of skip N2 is lymphatic flow from the lung directly to the mediastinum through the pleura [27]. Radical segmentectomy for patients with skip N2 metastasis has the possibility that micro cancer cells remain in pleural lymphatic ducts. Therefore, a preoperative or intraoperative predictive factor for skip N2 metastasis is necessary to choose adequate surgical resection.

Skip metastasis to mediastinal lymph nodes has been reported to occur in 20 to 40% of patients with N2 NSCLC [4,27,28]. In our study, the 5-year survival rate for skip N2 patients was even higher than that in other previous reports [17-22], which was because these previous reports included many patients with large-sized tumor (tumor diameter >3 cm) [18,20-22]. In addition, 75% of skip N2 patients had single-station disease, which was more frequent than the other reports [21,22] and affected this discrepancy. In several reports, clinicopathological factors were analyzed in patients with skip N2 metastasis. Skip N2 metastasis was more frequent with tumors in the upper lobes than the lower lobes [17,18], in right-sided lesions than left-sided lesions [21], and in cases of squamous cell carcinoma than in cases of adenocarcinoma [21,22]. In our study, there were no significant differences between pN0 and skip N2 patients in tumor side, location, or histology. Small-sized NSCLCs are heterogenous, including pure GGO, GGO with small consolidation and real consolidation. The proportion of GGO area on CT has been reported as a predictor of lymph node metastasis. There has been shown to be no lymph node metastasis in patients with c-stage IA adenocarcinoma with more than 50% proportion of GGO [29]. In addition, 98.7% of patients with c-stage IA NSCLC with less than 25% consolidation of the maximum tumor diameter showed pathological non-invasiveness [30]. In our study, the patients with c-stage IA NSCLC with more than a 75% proportion of GGO never exhibited skip N2 metastasis, and those with a 50 to 75% proportion of GGO occasionally exhibited skip N2 metastasis, as shown in Table 3.

Pathological factors such as pleural invasion [31] and tumor size [18] have also been reported to be associated with skip N2. There were no significant associations between skip N2 metastasis and surgical or pathological PL factor or tumor diameter in this study. One mechanism of skip N2 is pleural lymphatic flow [27], and ly and v factors have been reported to predict lymph node metastasis in NSCLC [32]. Therefore, we investigated whether distance to pleura or intersegmental plane, ly factor, or v factor were important predictors of skip N2 metastasis. Our data support distance to pleura, ly factor, and v factor as risk factors for skip N2 metastasis as shown in Table 3. Eight of twelve patients with skip N2 metastasis had peripheral lung cancers located close to the pleura (distance ≤5 mm), and eleven of twelve were positive for either ly or v factor. The only case of skip N2 that was close to the pleura and was negative for both ly and v factors was the largest tumor in the group (30 mm). Although ly and v factors were significantly associated with skip N2, it is important to note that these factors cannot be assessed preoperatively or intraoperatively. In our study, serum SLX concentration was the only useful preoperative or intraoperative test to help predict skip N2.

SLX is a carbohydrate antigen adhesion molecule that has been used as a tumor marker for carcinoma of many organs, including the lungs [33]. SLX plays an important role in cell-cell recognition and is therefore thought to be associated with the metastatic ability of cancer cells. In the case of lung cancer, we have reported that high serum concentrations of SLX are predictive of lymph node metastasis, postoperative recurrence, and poor prognosis in patients with NSCLC [34-36]. Several authors have reported that SLX is predictive of distant metastasis in patients with primary lung cancer [37-39]. As for other tumor markers, high serum CEA has also been reported to be a predictive factor for lymph node metastasis in patients with small-sized adenocarcinoma of the lung [40]. Although the AUC for SLX was 0.710, which was higher than that for CEA (0.611, *P* = 0.227) or for CYFRA21-1 (0.507, *P* = 0.106), results of multivariate logistic regression analysis showed serum SLX concentration was an independent predictive factor for skip N2 in patients with c-stage IA NSCLC. The calculated optimal cutoff point for serum SLX concentration in this study (21.4 U/mL) was lower than the accepted cutoff for cancer screening (38.0 U/mL). We propose that the prognosis cutoff value should be used to predict skip N2 metastasis rather than the diagnosis cutoff value.

## Conclusions

We found that serum SLX concentration was an independent predictive factor for skip N2 in c-stage IA NSCLC. Skip metastasis is common in NSCLC patients with high serum SLX, and lobectomy with complete dissection of hilar and mediastinal lymph nodes should remain the standard surgical procedure for these patients. Preoperative serum SLX levels have the possibility to change the present surgical procedure of segmentectomy for patients with c-stage IA NSCLC.

## Abbreviations

AUC: Area under the curve; CEA: Carcinoembryonic antigen; c-stage: Clinical stage; CT: Computed tomography; CYFRA21-1: Cytokeratin 19 fragment; GGO: Ground-glass opacity; ly factor: Lymph vessel invasion factor; NSCLC: Non-small cell lung cancer; PET: Positron-emission tomography; pN0: No pathological lymph node metastasis; pN1: Patients with hilar or interlobar lymph node metastasis; pPL factor: Pathological pleural invasion factor; ROC: Receiver operating characteristic; SLX: Sialyl Lewis X; sPL factor: Surgical pleural invasion factor; v factor: Venous invasion factor.

## Competing interests

The authors declare no competing interests.

## Authors’ contribution

NI, KC, SH, and HI participated in data acquisition. SM, SS, and NN participated in the conceptualization, preparation, and editing of the manuscript. HK drafted the manuscript. All authors read and approved the final manuscript.
